# Music Composition and Emotion Recognition Using Big Data Technology and Neural Network Algorithm

**DOI:** 10.1155/2021/5398922

**Published:** 2021-12-16

**Authors:** Yu Wang

**Affiliations:** Zhoukou Vocational and Technical College, Henan, Zhoukou 466002, China

## Abstract

To implement a mature music composition model for Chinese users, this paper analyzes the music composition and emotion recognition of composition content through big data technology and Neural Network (NN) algorithm. First, through a brief analysis of the current music composition style, a new Music Composition Neural Network (MCNN) structure is proposed, which adjusts the probability distribution of the Long Short-Term Memory (LSTM) generation network by constructing a reasonable Reward function. Meanwhile, the rules of music theory are used to restrict the generation of music style and realize the intelligent generation of specific style music. Afterward, the generated music composition signal is analyzed from the time-frequency domain, frequency domain, nonlinearity, and time domain. Finally, the emotion feature recognition and extraction of music composition content are realized. Experiments show that: when the iteration times of the function increase, the number of weight parameter adjustments and learning ability will increase, and thus the accuracy of the model for music composition can be greatly improved. Meanwhile, when the iteration times increases, the loss function will decrease slowly. Moreover, the music composition generated through the proposed model includes the following four aspects: sadness, joy, loneliness, and relaxation. The research results can promote music composition intellectualization and impacts traditional music composition mode.

## 1. Introduction

With rapid economic development, Chinese people are expecting a higher quality of spiritual life. Particularly, under diversified entertainment industries, music, as a kind of social ideology, can cultivate people's sentiment, regulate their emotions, and are of great practical significance. Meanwhile, music can encourage new ideas and brilliant lifestyles, and it has a strong infection. Streets and shopping centers are full of music rendering, giving people passion and joy [1]. Music has always been popular with the masses. Since ancient times, composers have tried new methods and techniques to meet people's needs. Today, under the Internet era, short-video platforms, the animation industry, and video games are attracting more and more users, in which extraordinary amounts of original music works are needed. Yet, high-quality music composition and production usually cost much time and resources, which has posed great challenges to meet users' personalized music demands [2]. With the development of the Internet and big data technology, a music composition can be automatically generated through an intelligent computer system, thereby greatly improving the vitality of music composition and encouraging music composers' inspiration for top-quality music composition. Additionally, the ever-increasing music works should be classified and managed scientifically. Significantly, specific algorithms can be used for music composition, and ideas of the mainstream intelligent music composition algorithm are to utilize the structural thinking of a selected music composition for new works, which can minimize the interference of human factors [3]. Under the rapid socio-economic development, music works are changing in multidimensions with subtlety, which are reflected in several aspects: polyphony, track structure, harmony, melody speed, and rhythm. Moreover, different types of music can be generated through a different combination of these factors, such as rap, classical music, and rock music [4]. Presently, based on the intelligent computer music composition, some technical methods have been put forward for practical applications, which include the Genetic Algorithm (GA), music grammar, and Neural Network (NN) algorithm [5].

Under the background of big data, this paper realizes the generation of the music composition and emotional recognition of composition content through the NN algorithm. It is hoped that this research can further promote the intellectualizations of the music composition industry and help musicians generate better music tracks. Innovatively, four NN algorithms are combined to implement an automatic music composition generation model, which can well ensure the excellency and integrity of the generated music composition, greatly improve the writer's musical creativity, reduce the creative threshold of nonprofessionals, and assist the composer to explore new creative ideas.

## 2. Related Works

In the context of big data, the NN algorithm has been widely applied in various fields. However, the research of the application of NN in music composition is becoming one heated topic and is of great significance due to relatively small existing studies.

Metcalf integrated space into music and expanded the concept of music electrocardiogram (ECG) through the combination of the selected composition methods related to creative design and audience communication with other contemporary music examples and trends [6]. Hervé et al. found that the extraction of semantic memory and episodic memory was completed by different NN. However, these results were obtained through language and visuospatial materials. The purpose was to determine the neural basis of semantic and plot components of music using familiar and nonfamily melodies [7]. Jin et al. studied music composition and found that the automatic music composition model could greatly reduce the music production cost and the threshold of nonprofessional composition, thereby improving the music composition efficiency. Consequently, an intelligent music creation NN model was proposed to automatically generate a specific style of music. The advantage of the proposed model was its innovative structure: the music sequence was obtained through the actor's long-short memory, and then the probability of the sequence was determined through a reward-based process and was fed back to improve the performance of the music works. The rules of music theory were introduced to constrain the style of generated music [8]. Wang et al. proposed a new end-to-end Deep Neural Network (DNN) model for music automatic annotation. The model effectively integrated various complementary music representations to complete music representation learning, structure modeling, and label prediction. Firstly, the model learned information description with attention convolution network and recursive network from Mel spectrum and original music waveform and described the time-varying structure embedded in the described sequence. Then, the correlation between the two presentation channels was captured as a supplementary music description using the dual state Long Short-Term Memory (LSTM) network. Finally, the model aggregated the music description sequence into a whole and embedded it through a self-focusing multiweight mechanism to adaptively obtain the summary information of music for label prediction [9]. Kim found that scenes in music programs should be constantly edited to maximize audience immersion. Music program scene editing was developed through the professional knowledge of the television Program Director (PD). Therefore, a music program scene editing algorithm was proposed, which determined the size of the shot by measuring the pitch contour of the song and evaluated the psychological distance between the singer and the audience [10]. Yan et al. suggested a cognitive NN based on Takagi Sugeno (T-S) model to train the network weights with improved GA. The membership function parameter adjustment strategy was combined with the momentum method and learning rate-adaptive adjustment, and the results showed that the combined method could be applied to the music recognition system, and the recognition accuracy of the algorithm was higher than other algorithms with good robustness [11]. Gao and CAI proposed that with the help of Geographic Information System (GIS) technology, designers could better optimize the urban regional function positioning and urban function zoning in the study of big data and GIS [12].

To sum up, the above research indicates that the application of big data and NN in the field of music is maturing. Meanwhile, the automatic music composition and recognition of composition contained in the above studies are realized through the NN model, which has a crucial impact on both the quality of music works and the recognition accuracy. Here, the search theme and content are based on previous achievements, and the purpose is to explore the application of big data technology and NN algorithm in the music composition and emotion recognition of composition content.

## 3. Design of the Music Composition Algorithm

### 3.1. Music Composition Style

With social progression and the improvement of people's living standards, culture, and art are developing steadily, and music, in particular, is developing from many aspects, such as melody, rhythm, harmony, polyphony, structure, form, and arrangement. The style of music often changes continuously over time, so the music style often overlaps with those of other periods. Technically, there are no strict music style division standards, but generally, music can be categorized as pop music and classical music [13].

#### 3.1.1. Classification of Classical Music

Classical music has influenced several generations with its profound historical connotation, and it reflects people's feelings in different historical periods through its inherent emotions and humanistic feelings and has gained its stance in modern fast-food entertainment culture. Classical music can be defined in a broad sense and a narrow sense. In a broad sense, classical music has been developing for over nine centenaries, and it originates from modern European and Western culture, including Western secular music and traditional Church music [14]. In a narrow sense, classical music is also called Vienna classical music, which refers to the music works led by Beethoven and Mozart in the 18th century. Classical music has a lasting charm because of its structure, rigorous form, and full emotion, and it has experienced a long-term development. Particularly, the Renaissance age has witnessed the fall of the Church power, as well as the political turbulence, poor social disorder, and the emergence of the bourgeoisie in Europe. Consequently, some aspiring young musicians begin to use their own way to publicize some ideas, thereby giving birth to the traditional major key and minor key. With the stabilization of Europe in the Baroque period, the development of music has entered a new stage, and then four-part harmony and chord with words in classical music are born. When the late Baroque period arrives, the main forms of music have changed significantly. At that time, it is more dazzling, rich, and free in content compared with traditional religious music. Meanwhile, many excellent composers like Bach and Handel are born. The end of the Baroque period symbolizes the advent of the period of Vienna classical music, whose music form and music structure are dominated by those of the Baroque period but are integrated with people's emotional factors more, and the content of music becomes more abundant [15].

The year 1820 has seen the birth of romantic music. At that period, music is closely correlated with people's life and focuses on the emotional expression of the human spirit in the world. In terms of creation, the form of music is more abundant, and the emotion is more popular. Importantly, Chopin and Will have made great contributions to this period, and Tchaikovsky and Wagner have reached their heyday, thus establishing a good foundation for the development of classical music. In the 19th century, Impressionist music represented by Debu and Webern come into being. Electronic music technology has developed rapidly after the Second World War, the communication between countries has been frequented, the music forms become more open and diverse, the music theory gets matured, and some obscure music forms are also created, such as silent music, differential music, and vocal music.

#### 3.1.2. Pop Music Classification

Compared with other music, pop music is more distinctive. Before 1980, the types of pop music are monotonous, including country music, jazz, and blues. After 1980, with the rapid development of network multimedia, the music style has changed greatly. During this period, the blue note is also known as blues. Blues is first created by black people in the second half of the 19th century to express their feelings, and the music style of blues has not been fixed until the 20th century. In terms of content, blues contain the cry of the vast African fields, as well as the Christian hymns. The main style of blues is expressed using string or grade, and its main form is divided into 8 bars, 12 bars, and 16 bars, of which the most frequently used is 12 bars [16].

Jazz is born in the early 20th century and is featured by fast rhythm and full power, which is very characteristic but not out of order, thereby gaining love and respect from many musicians and young people. Compared with the blues, jazz is more abundant, including American music, African tribal music, and European music, as well as pop music and folk music. Because jazz has a very high form of change, its content also includes all areas of life, which is in line with the mainstream development of society. So far, the development of jazz is the best.

In 1920, a new type of music has emerged: country music, which is born in the southern United States. In terms of composition content, it mainly expresses the living environment of the black people at that time and their yearning for a better life. The early development of country music depends mainly on the violin, harmonica, guitar, and other instruments to accompany the performer's singing. In terms of musical expression: country music is composed of simple structure, fluent content, and catchy-and-sweet lyrics, and they are mostly ballad style, two-part form, or trilogy. Notably, there is a big difference between country music and urban pop music. Country music is more stable in rhythm and has a strong rural flavor. In terms of the theme of music creation, country music has the following eight ways: God and country, love, cowboy humor, regional pride, music, lovelorn, rural lifestyle, and family.

### 3.2. Artificial Neural Network (ANN)

Nowadays, in the era of big data, ANN has become an important information processing method, which can accurately transfer information between neurons. ANN algorithm simulates the transmission principle of neurons using the functional mechanism of the human brain. Consequently, a new NN algorithm, namely, ANN, is proposed from the perspective of NN signal processing. The model is abstract and can be mapped to form different NN models using different functions [17].

#### 3.2.1. Perceptron

Perceptron is a NN model with a relatively simple structure based on Support Vector Machine (SVM), but it can only deal with the linear problem of binary classification. The perceptron can simulate the dendrites, cell bodies, and synapses between neurons. While the specific state of the cell body itself is still affected by the signal sent by the previous neuron and the current synapse state, if the amount of information received from the cell exceeds the specified threshold value, the cell body will be stimulated and generated by the electrical signals transmitted by the axial and synaptic signals to the next neuron. Similarly, the process will repeat itself on each cell body [18], as shown in Figure 1.

Figure 1 shows the single-layer perceptron structure to simulate the process, in which *x*_1_, *x*_2_, and *x*_3_ are the three inputs of the model, and *w*_1_, *w*_2_, and *w*_3_ are the corresponding weights. After the weighted summation of the input and the weights, the final result *y* is output through the activation function mapping.

#### 3.2.2. NN Structure

The brain has a complex structure and is composed of many neurons. If each perceptron represents a neuron in the brain, then a NN can be built through mutual connections and combinations of plenty of perceptrons, as shown in Figure 2. The structure of NN includes the output layer, hidden layer, and input layer; the hidden layer can assign different weights to different perceptron according to their recognition ability, and the output layer can output the processed data/signal [19, 20]. The NN model can handle nonlinear problems. The multiclassification problem can be processed using the NN model with an output layer of two neurons.

The NN updates information through forwarding propagation and backward propagation.

#### 3.2.3. Recurrent Neural Network (RNN)

RNN is a ring-type network structure, in which the output of the neural unit is related to the input at the current moment as well as to the value at the previous moment. This structural feature can be used for timing problems [21], as shown in Figure 3.

The calculation method of RNN can be expressed as in the following equations:

(1) $$\begin{array}{c} O_{i}=g\left(V\cdot S_{i}\right), \end{array}$$

(2) $$\begin{array}{c} S_{i}=f\left(U\cdot X_{i}+W\cdot S_{i-1}\right). \end{array}$$

In the above equations, *X* represents the input data, *U* denotes the weight vector between the input layer and the hidden layer, *S* indicates the hidden layer data, and *V* is the weight vector between the hidden layer and the output layer. Meanwhile, *O* stands for the output data, and *W* is the weight vector between the hidden layer and the hidden layer.

#### 3.2.4. LSTM Network

The hidden layer of LSTM contains three gate structures: output gates, forget gates, and input gates. The three gates can realize *U* control of information transmission. In each gate, there is a dot multiplication operation and a Sigmoid layer. The output range of the Sigmoid layer is [0, 1], which can describe how much information is passed in each part, where 0 means no pass and 1 means all pass [22].

(1) The input layer information *C*_*t*_ is calculated using equation (3), where *W*_*ij*_ represents the weight vector between the input data and the hidden layer, *W*_*jc*_ denotes the output weight at the previous moment, and *b*_*c*_ indicates the offset.
  (3) $$\begin{array}{c} C_{t}=\tanh\left(w_{ij}x_{t}+w_{jc}C_{t-1}+b_{c}\right). \end{array}$$
(2) The input gate *i*_*t*_ is calculated using equation (4), where *W*_*xi*_ represents the weight between the input gate and the input information, *w*_*ih*_ stands for the weight between the input gate and the output at the previous moment, *w*_*ci*_ denotes the weight between the input gate and the cell at the previous moment, and *b*_*i*_ is the offset.
  (4) $$\begin{array}{c} i_{t}=\psi \left(w_{xi}x_{i}+w_{hi}h_{i-1}+w_{ci}c_{t-1}+b_{i}\right). \end{array}$$
(3) Similarly, the forget gate is calculated using the following equation:
  (5) $$\begin{array}{c} f_{t}=\psi \left(w_{xf}x_{t}+w_{hf}h_{t-1}+w_{cf}c_{t-1}+b_{f}\right). \end{array}$$
(4) The state value in the cell is calculated using the following equation:
  (6) $$\begin{array}{c} c_{t}=f_{t}⊗c_{t-1}+i_{t}⊗c_{t}. \end{array}$$
(5) The output gate state value is calculated using the following equation:
  (7) $$\begin{array}{c} O_{t}=\psi \left(w_{xo}x_{t}+w_{ho}h_{t-1}+w_{co}c_{t-1}+b_{o}\right). \end{array}$$
(6) Finally, the output of the LSTM network is obtained using the following equation:

(8) $$\begin{array}{c} h_{t}=o_{t}⊗\tanh\left(c_{t}\right). \end{array}$$

#### 3.2.5. Convolutional Neural Network (CNN)

CNN is a multilayer network structure composed of a convolutional layer, pooling layer, and fully connected layer [23]. After the convolution operation, the convolutional layer can select the local features of the upper layer. During image processing, the convolution operation is essentially the image filtering process using the convolution kernel. The convolution operation of the image is shown in the following equation:

(9) $$\begin{array}{c} f\left(x,y\right)*w\left(x,y\right)=\overset{a}{\underset{s=-a}{\sum }}\overset{b}{\underset{t=-b}{\sum }}w\left(s,t\right)f\left(x-s,y-t\right). \end{array}$$

In equation (9), *f* (*x*, *y*) represents the point gray value of the selected image in a coordinate system, *w*(*x*, *y*) represents the convolution kernel, and (*a*, *b*) represents the size of the convolution kernel.

### 3.3. Music Composition Algorithm Based on Music Composition Neural Network (MCNN)

Here, a new MCNN structure is proposed from the perspectives of big data and music theory creation. Network model training: LSTM generation network is pretrained by inputting a classical music database in MIDI format, initial notes are set to randomly generate music, the generated music is collected, and a music generation sample database is constructed and marked as 0, while the training dataset is marked as 1. At the same time, a binary classification model has been implemented, and CNN is pretrained. In the process of music sequence generation, the music sequence is generated by the LSTM network based on the initial notes setting. Different from the training model, in the MCNN model, the generated music data tag is set to 1 and outputs through CNN. The output binary classification discrimination probability is *P*_(CNN)_, and the Reward function is formed through the weighted calculation with music theory rules, and the LSTM network parameters are updated and adjusted through Reward function calculation. The music generation model uses the idea of the chess game. CNN hopes to identify the label 0 of the generated music, and the generation model tries to make the generated music and training samples have a greater degree of confusion through the optimization of the Reward function to make the recognition output probability of the classification network CNN closer to 0.5, that is, there is no difference between the generated samples and training samples, to get music with similar style and theme as the training sample.

#### 3.3.1. Music Composition Sequence Generation

Music is a kind of time sequence. The LSTM network is used to generate music sequences. The LSTM has a special timing memory function [24, 25]. Based on the common multilayer Backpropagation neural network (BPNN), LSTM adds the horizontal connection between the units of the hidden layer. Through a weight matrix, the previous information can be connected to the current task. Let the training sequence be the input sequence *X*_in_ = (*x*_1_, *x*_2_,…, *x*_*T*1_), the output *Y*_out_ = (*y*_1_, *y*_2_,…, *y*_*T*2_), and *T*1 and *T*2 are the input and output sequence lengths. Then, the generated sequence *y*_*t*_ based on the LSTM network can be obtained by iterating the following equation:

(10) $$\begin{array}{c} s_{t}=f\left(x_{t},S_{t-1}\right), \end{array}$$

(11) $$\begin{array}{c} y_{t}=W_{\text{out}}\times S_{t}, \end{array}$$

where *f* is the activation function, and *W*_out_ ∈ *R*^*n*×*m*^ belongs to the weight matrix. At the same time, *W* is initialized and then updated iteratively to achieve better performance.

#### 3.3.2. Reward Function and Similarity Probability

According to the basic criteria of music creation, a music evaluation function, Reward, is proposed to supervise and adjust music composition in real time, thus making up the deficiency of a single LSTM network, creating music even closer to the composer's creative thinking, and ultimately, meeting the needs of the audience [26, 27]. The Reward function can evaluate the quality of the music generated by the LSTM network, feedback the evaluation results to the generated network, and adjust the parameters of the LSTM network.

CNN has good classification performance in pattern recognition, and it extracts the image features using convolution kernel and then outputs the classification results through the Softmax layer. In the systematic updating and optimization of the network, to make the actual music composition samples close to the training samples, a CNN binary neural network model is established [28]. Here, the generated music composition sample set is marked with the number 1. The discriminant probability is output through the CNN to compare the similarity between the generated music composition samples and the training samples of music composition. LSTM can transform the MIDI (Musical Instrument Digital Interface) note sequence into the piano roll and input it into the CNN model [29]. Every cycle will generate a music sequence, and every time the music sequence is generated, the file format is transformed, and the CNN neural network model outputs the similar probability *P*_(CNN)_.

(12) $$\begin{array}{c} P_{\left(\text{CNN}\right)}=\left\{\begin{array}{cc} 0, & \text{for }t<T,\\ D_{\phi }\left(\alpha_{1:T}\right)-0.5, & \text{for }t=T. \end{array}\right) \end{array}$$

In MCNN, the updating process of the LSTM network and Reward network is shown in Figure 4 during the continuous iteration of weight parameters. First, strategy *π* is defined: *S* to *A* is the mapping from state space to action space. At time *t*, the generation (LSTM) network selects an action according to the policy *π* in the current state *s*_*t*_, generates a note, executes the action, transfers to the state *s*_*t* + 1_, and feeds back the Reward *Q* of the action. The Reward network evaluates the advantages and disadvantages of the action strategy by calculating the cumulated Rewards of the action sequence, updates the LSTM network parameters, and adjusts the sequence generation strategy *π* to obtain a larger Reward.

The Reward network consists of the Q-target network and Q-action network. The Q-target network is copied from the Q-action network every *N* step, and its value function reads as follows:

(13) $$\begin{array}{c} J\left(s,\alpha ,\theta_{v}^{-}\right)=R+\gamma \max Q\left(s^{\prime },\alpha^{\prime },\theta_{v}^{-}\right)+V\left(s;\theta_{v}^{-}\right), \end{array}$$

where *R* is the Reward under action *α* in the state *s*. *s*′ indicates the next state after action *s*′, and *α*′ denotes the next action. *θ*_*v*_^−^ means the target value network parameter. *γ* stands for the discount factor, and *v* is the state value function. Under the Monte Carlo tree algorithm, in the state *s*, *N* and *α* actions are sampled based on strategy *π*, and the mean Reward *v* is obtained. The value of V can be calculated according to the following equation:

(14) $$\begin{array}{c} v=\frac{1}{N}\sum_{n=1}^{N}R\left(s,\alpha_{n},\theta_{v}^{-}\right). \end{array}$$

In the Reward network, the loss function of the action network and the target network is calculated as

(15) $$\begin{array}{c} \sigma \left(\theta_{v}\right)=\lambda \left(J\left(s,\alpha ,\theta_{v}^{-}\right)\right)-Q\left(s,\alpha ,\theta_{v}\right), \end{array}$$

where *θ*_*v*_ is the target value network parameter, and *λ* represents the discount factor of the target function value.

### 3.4. Music Emotion Feature Extraction

Here, the emotion features of the audio signal are extracted from the time domain, frequency domain, time-frequency domain, and nonlinearity, as shown in Figure 5.

#### 3.4.1. Pitch Frequency

In Mandarin, different intonations of the same word may have different meanings, and different tones correspond to different pitch tracks. Pitch is one major parameter of acoustics. The pitch frequency plays an important role in sound signal analysis, so it is often used in speech recognition and audio analysis.

#### 3.4.2. Short-Term Energy

Short-term energy can distinguish voiced and unvoiced sounds. In the mathematical calculation, the short-term energy can be obtained through the window function setting. If *x*(*l*) is set as the audio time-domain signal, *ω*(*m*) is set as a window function, then the *n*th frame signal *x*_*n*_(*m*) can be obtained using the frame division and window processing, as shown in the following equation:

(16) $$\begin{array}{c} x_{n}\left(m\right)=\omega \left(m\right)x\left(n+m\right),\;0\leq m\leq N-1, \end{array}$$

(17) $$\begin{array}{c} \omega \left(m\right)=\left\{\begin{array}{cc} 1, & m=0∼\left(N-1\right),\\ 0, & m=\text{else}. \end{array}\right) \end{array}$$

#### 3.4.3. Short-Time Zero-Crossing Rate

The number of times the audio waveform signal passes through the time axis is called the short-time zero-crossing rate, which can also be used to distinguish voiced and unvoiced sounds. The unvoiced sound generally appears in the high-frequency band, and the zero-crossing rate is often larger. On the contrary, the voiced sound generally appears in the low-frequency band, and the zero-crossing rate of voiced is smaller. The short-time zero-crossing rate *Z*_*n*_ of the *n*th frame signal *x*_*n*_(*m*) can be obtained using the following equation:

(18) $$\begin{array}{c} Z_{n}=\frac{1}{2}\sum_{m=1}^{N-1}\left|\mathrm{sgn}\left(x_{n}\left(m\right)\right)-\mathrm{sgn}\left(x_{n}\left(m-1\right)\right)\right|. \end{array}$$

In the equation below, SGN represents the sign function.

(19) $$\begin{array}{c} \mathrm{sgn}\left(x\right)=\left\{\begin{array}{cc} 1, & x\geq 0,\\ -1, & x<0. \end{array}\right) \end{array}$$

#### 3.4.4. MFCC (Mel Frequency Cepstral Coefficient)

The Mel filter bank is similar to the human cochlea in the model, which can respond positively to the frequency signals of various sounds. In the actual environment, human sound perception differs greatly under different sound frequency ranges [30]. When the frequency of the received sound signal is lower than 1,000 Hz, the sound perception and signal frequency are a linear relationship; by comparison, when the frequency of the received sound signal is higher than 1,000 Hz, the relationship between the two is logarithmic, as shown in the following equation:

(20) $$\begin{array}{c} \text{Mel}\left(f\right)=25951\left(1+\frac{f}{700}\right). \end{array}$$

In the above equation, *f* represents the actual frequency, and Mel (*f*) denotes the frequency perceived by the human ear.

## 4. Analysis of Experimental Results

### 4.1. Analysis of the Result of Music Composition

Figure 6 shows the music spectrum.  Figure 7 illustrates the impact of different iteration times on the results.

Figure 6 suggests that the more LSTM cells in the hidden layer are, the stronger the LSTM network can learn abstract data features and narrow the gap between the target value and the predicted value. At the same time, the dimension of the hidden layer also seriously impacts the experimental results: when the number of hidden layers increases, the NN calculation will spike. The continuous iteration of weight parameters has a great impact on the generation results of music composition and the loss function. The results are shown in Figure 6. The data variation in Figure 6 imply that the greater the number of iterations is, the more the number of weight parameter learning and adjustment is, which can somehow improve the model accuracy of the model *t*. And with the increase of the number of iterations, the decline of loss function slows down gradually. Inevitably, excessive iterations will also bring more computation.

### 4.2. Test Results of MCNN Algorithm

Figure 8 illustrates the time-domain waveform of training samples and generated samples under the MCNN algorithm.

Figure 8 demonstrates that the frequency distribution of the changing waveform of music composition generated by the MCNN algorithm and the training sample waveform is similar, so the MCNN algorithm can learn the internal structure of training samples well.  Figure 9 illustrates the comparison results of three music composition algorithms, VAE-GAN, GAN, and RL-RNN.

Figure 9 implies that, compared with other algorithms, the music composition generated by the proposed MCNN algorithm can achieve a high-sample pass rate, which is far higher than GAN and VAE-GAN and slightly better than the RL-RNN algorithm. Therefore, the music generated by the MCNN algorithm can ensure the integrity of music composition. The music composition model built with big data learning and music composition has higher practicability.

### 4.3. Music Emotion Recognition Test

Figure 10 shows the validity test of music emotion feature extraction and classification algorithms.

Figure 10 displays that the spectrogram characteristics, frequency-domain characteristics, linear Hurst parameters, and time-domain characteristics analyzed here play an important role in music composition. Meanwhile, in terms of music classification and recognition, the decision tree with poor classification performance should be reduced. The music composition of automatic generation consists of four aspects: sadness, joy, loneliness, and relaxation, in which, sentimental music accounts for more.

## 5. Conclusion

Here, the music composition and emotion recognition of composition content is analyzed using big data technology and the NN algorithm. Based on the analysis of RNN, LSTM, and CNN, an automatic music composition model based on MCNN is established. Meanwhile, the emotion features are extracted and recognized through the four aspects of music composition content: time-frequency domain, frequency domain, nonlinearity, and time domain. The results show that the more the number of LSTM cells in the hidden layer structure is, the stronger the learning ability of the LSTM network is for abstract data features, and the narrower the gap between the target value and the predicted value is. The frequency distribution of the music composition generated by the MCNN algorithm is similar to that of the training samples, thus proving that the MCNN algorithm can learn the internal structure of the training samples well. Additionally, the automatically generated music includes the following four aspects: sadness, joy, loneliness, and relaxation, in which, sentimental music accounts for more. Still, there are some limitations. Increased iterations will bring a huge amount of calculation, the increase of the number of hidden layers also multiplies the calculation of the model. Therefore, in future research, a more efficient algorithm should be chosen to reduce the computational works of the model.

## Figures and Tables

**Figure 1:** Perceptron structure.

**Figure 2:** Network structure diagram. (a) Neural network structure; (b) multiclassification network structure.

**Figure 3:** RNN network structure. (a) Structure diagram; (b) simplified structure diagram.

**Figure 4:** MCNN update process.

**Figure 5:** Emotion features of music.

**Figure 6:** Influence of different LSTM cells on experimental results (a/b/c/d represent the influence of different LSTM cells on experimental results, respectively). (a) Training dataset. (b) Hidden-layer128.wav. (c) Hidden-layer512.wav. (d) Hidden-layer1024.wav.

**Figure 7:** Influence of different iteration times on the experiment (a/b/c indicate the influence of different iteration times on the results, respectively; d: influence of iteration times on loss). (a) Epochs1000.wav. (b) Epochs2000.wav. (c) Epochs3000.wav. (d) The influence of iteration number on loss number.

**Figure 8:** Time-domain waveforms of training samples and generated samples. (a) The waveform of the original music. (b) The waveform of the generated music.

**Figure 9:** Pass rate of four music composition algorithms (A: SeqGAN; B: VAE-GAN; C: RL-RNN; D: MCNN).

**Figure 10:** The validity test of music emotion feature extraction and classification algorithms; (a) validity test of classification algorithm; (b) emotion recognition; A: spectrogram; B: time-domain characteristics; C: frequency-domain characteristics; D: multifeature fusion + DERF; E: multifeature fusion + RF; F: multifeature fusion + SVM; G: multifeature fusion + BP; 1: sadness; 2: joy; 3: loneliness; 4: relaxation.

## Data Availability

The data used to support the findings of this study are available from the author upon request.
